# Effects of Data Augmentation with the BNNSMOTE Algorithm in Seizure Detection Using 1D-MobileNet

**DOI:** 10.1155/2022/4114178

**Published:** 2022-12-19

**Authors:** Peiling Zhang, Xuan Zhang, Ankang Liu

**Affiliations:** School of Physics and Electronic Information, Henan Polytechnic University, Jiaozuo 454000, China

## Abstract

Automatic seizure detection technology has important implications for reducing the workload of neurologists for epilepsy diagnosis and treatment. Due to the unpredictable nature of seizures, the imbalanced classification of seizure and nonseizure data continues to be challenging. In this work, we first propose a novel algorithm named the borderline nearest neighbor synthetic minority oversampling technique (BNNSMOTE) to address the imbalanced classification problem and improve seizure detection performance. The algorithm uses the nearest neighbor notion to generate nonseizure samples near the boundary, then determines the seizure samples that are difficult to learn at the boundary, and lastly selects seizure samples at random to be used in the synthesis of new samples. In view of the characteristic that electroencephalogram (EEG) signals are one-dimensional signals, we then develop a 1D-MobileNet model to validate the algorithm's performance. Results demonstrate that the proposed algorithm outperforms previous seizure detection methods on the CHB-MIT dataset, achieving an average accuracy of 99.40%, a recall value of 87.46%, a precision of 97.17%, and an F1-score of 91.90%, respectively. We also had considerable success when we used additional datasets for verification at the same time. Our algorithm's data augmentation effects are more pronounced and perform better at seizure detection than the existing imbalanced techniques. Besides, the model's parameters and calculation volume have been significantly reduced, making it more suitable for mobile terminals and embedded devices.

## 1. Introduction

Epilepsy is a chronic neurological condition caused by aberrant firing of nerve cells in the brain [1]. Epilepsy affects more than 50 million people globally, according to statistics, and the number is growing every year. Despite the fact that some individuals' illnesses can be controlled with medicines or surgery, roughly one-third of persons with epilepsy do not respond well to antiepileptic drugs (AEDs) or have no effective treatment, a condition known as refractory epilepsy [2]. Because of the human central nervous system's structural and functional complexity, aberrant discharges brought on by epileptic seizures can affect various parts of the cerebral cortex or subcutaneous layer. Rapid brain spread results in a variety of epileptic seizure symptoms as well as complex and diverse clinical presentations.

Epilepsy is currently one of the most common disorders, with irregular seizures, often accompanied by loss of consciousness, involuntary convulsions, increased heart rate, and elevated blood pressure [3]. If you are in a potentially risky location at this time, such as stairs or roadways, the patient is likely to get additional harm [4]. The recurrence of epileptic seizures puts refractory patients at long-term risk of developing epilepsy, which seriously affects their physical and mental health and quality of life. For such intractable epilepsy patients, the current commonly used treatment method is long-range video electroencephalography (VEEG) monitoring, which evaluates the development of the disease by observing the patient's clinical response and analyzing abnormal EEG waveforms during epileptic seizures [5]. However, this approach has drawbacks such as low work efficiency, uneven ward monitoring, high treatment costs, and an impact on patients' daily lives, making it unsuitable for long-term monitoring. Automatic epilepsy detection technology will provide a more efficient technique to increase epilepsy diagnosis efficiency [6, 7].

In order to focus on this problem, researchers are using deep learning techniques. Deep learning is currently being used for a wider range of tasks, such as image classification, object detection, and semantic segmentation. By using the region-growing algorithm and the improved genetic algorithm for segmentation and feature extraction, respectively, Kaluri and Pradeep [8] improved the recognition rate by about 10% compared with the existing methods in gesture recognition. In addition, in a follow-up study [9], they improved the region growing algorithm and used an adaptive genetic fuzzy classifier (AGFC) for feature extraction and recognition. They used a genetic algorithm with a fuzzy classifier to find out the optimal rules generated by the fuzzy classifier, and the final average recognition rate could reach 83%.

The rest of this paper is arranged in the following way: Section 2 outlines the related work about seizure detection. The proposed methods are detailed in Section 3.  Section 4 presents the analysis of the results and the necessary discussion. Finally, the conclusion and prognosis are included in Section 5.

## 2. Related Works

Many scholars have expressed interest in automatic seizure detection technology, and various seizure detection algorithms have been presented. Acharya et al. [10] first applied convolutional neural networks (CNNs) to the study of EEG signal analysis, implementing a 13-layer deep CNN algorithm to detect normal, preictal, and seizure categories. Ultimately, they achieved an average accuracy of 88.7%, a specificity of 90%, and a sensitivity of 95% on the Bonn dataset. However, its main drawback is the lack of a large EEG database. The proposed algorithm needs diverse data to achieve the best performance. Segundo et al. [11] processed electroencephalogram signals using the Fourier transform (FT), wavelet transform (WT), and empirical mode decomposition (EMD), respectively. Then, they used a two-layer CNN for feature extraction and classification. Although more than 95% accuracy can be obtained on the Bonn dataset, it is too single to use only one evaluation index. In addition, when combining all transforms, they obtained slightly better results but not statistically different from the best result obtained using individual transforms. Gundluru et al. [12] designed a deep learning model with principal component analysis (PCA) for dimensionality reduction, and the Harris Hawks optimization algorithm is used further to optimize the classification and feature extraction process. Finally, the specificity, precision, accuracy, and recall rate are very much satisfactory compared to the existing systems. Nevertheless, in the event of a low-dimensional dataset, the model's ability to perform well may be limited by the possibility of overfitting.

Nowadays, multichannel EEG signal detection is commonly used to improve the accuracy of seizure detection. For multichannel EEG signals, Jana et al. [13] studied the effectiveness of discrete wavelet transform (DWT) and EMD feature fusion on four different classifiers for seizure detection, and finally, the accuracy and F1-score reached more than 90%. Moreover, Diykh et al. [14] proposed a wavelet-based texture approach to detect seizures. They found that only 59 of the texture features can exhibit the abnormal increase in EEG amplitude and the spikes notable during a seizure and then designed an ensemble classifier method to realize automatic detection of neonatal seizure from multichannel EEG signals.

Due to the large memory requirements and a large amount of parameter calculation of traditional neural network models, it is difficult to run on mobile terminals and embedded devices. Therefore, lightweight neural networks emerge as the times require. Zhu et al. [15] predicted the feasibility of sudden death in epilepsy (SUDEP) using a lightweight CNN, proposed a baseline CNN model with a lightweight structure, and finally attained an area under the curve (AUC) of 0.72. Shelatkar et al. [16] applied their modified lightweight deep learning model to medical imaging. They applied YOLOv5's different variant algorithm on the Brats 2020 annotated dataset to detect brain tumor location and achieved accuracy rates of 82% to 92%. In recent years, some lightweight network structures have been proposed, such as GhostNet [17], ShuffleNet [18], and MobileNet [19], among which the MobileNet series is particularly effective and more representative. Silva et al. [20] used MobileNet combined with transfer learning for EEG analysis in the study of automatic diagnosis of alcoholism patients. They finally achieved 95.33% accuracy and 95.24% F1-score, far exceeding the performance of classical extractors, which also proves the superiority of MobileNet series.

However, existing studies focus mostly on new feature extraction and classification approaches, while the disparity between seizure and nonseizure data distribution remains a technological challenge. In fact, in long-term continuous EEG recordings, due to the contingency of seizures, the nonictal period is substantially longer than the ictal period [21]. If it is not processed, the discriminant decision is likely to be biased towards the majority classes, negatively impacting classification results. Therefore, data balance is crucial to improve epilepsy detection performance.

Recently, some studies on imbalanced epilepsy datasets have been undertaken to address this issue. Amin and Kamboh [22] combined random undersampling with AdaBoost to classify epilepsy signals. Although they achieved good results, they lost a lot of valid data, so undersampling was not an effective method. Alkanhal et al. [23] employed random sampling techniques to balance the proportion of data in ictal and nonictal periods and optimize the complexity of the network, which improved the sensitivity, specificity, and accuracy to a certain extent. However, they converted EEG signals into multispectral and temporal images, which inevitably lost some of their signature information. To increase the number of preictal EEG signals, Zhang et al. [24] performed signal segmentation and reorganization in the temporal domain, followed by a feature extraction method combining wavelet packet decomposition (WPD) and common spatial pattern (CSP), and finally CNN for classification. Their advantage in dealing with imbalances is that they produce real data. However, they disrupted the original arrangement and distribution order because they randomly selected training segments for series, which went against the original intention of seizure detection and could not be applied to the research and development of smart devices. Zhao et al. [25] utilized focal loss to redefine the loss function of the linear graph convolution network (LGCN) to deal with the data imbalance problem during seizure detection. Finally, the accuracy of 99.30% and F1-score of 98.73% were achieved on the CHB-MIT dataset. Haldar et al. [26] adopted the synthetic minority oversampling technique (SMOTE) and selective preprocessing of imbalanced data algorithm (SPIDER) for imbalanced data, together with the k-nearest neighbor (KNN) classifier to increase epilepsy detection performance. The experimental results are up to 95% accuracy and F1-score. Jiang and Zhao [21] combined the SMOTE algorithm with the undersampling TomekLink technique to balance the data set, and compared with the previous five unbalanced processing methods, the sensitivity and accuracy reached 86% and 94%, respectively. However, there was no detailed analysis in the data preprocessing part, and the performance of individual patients in the experimental results was still very poor, and some even had a sensitivity lower than 60%. Kumar et al. [27] evaluated the empirical performance of six classifiers on seven different category balancing techniques on five imbalanced clinical datasets according to the imbalance problem in clinical datasets so as to achieve the purpose of data augmentation. Relatively speaking, SMOTEEN with KNN provided the highest accuracy, recall, precision, and F1-score over all the machine learning techniques all others for the BCD dataset. Gao et al. [28] built a generative adversarial network (GAN) to perform data augmentation to produce EEG data during seizures, which could be used to form a more balanced training set. Then, they designed a pyramidal one-dimensional CNN (1D-CNN) to process 1D EEG signals and achieved good results on three different epilepsy data sets.

In addition to the above-imbalanced treatment methods, there are also random oversampling (ROS) and improved borderline-SMOTE (BLSMOTE) [29] and SVM SMOTE algorithms based on SMOTE. Chen et al. [30] introduced the BLSMOTE algorithm to obtain a more balanced EEG feature set. Then, the 1D-CNN model is trained for three-classification in two dimensions of emotional valence and arousal, and finally, the average accuracy rate of 32 subjects on valence and arousal are 97.47% and 97.76%, respectively. It proves the validity of the idea of “data augmentation + classification,” which is very helpful for the research of our paper. However, there are some flaws in the BLSMOTE algorithm. It will cause the model to overlearn boundary data features, diminishing the influence of other data on the model, and it will be unable to effectively distinguish noise samples. Furthermore, in some cases, the method does not detect seizure samples at borderline locations [31]. In addition, although GAN can generate clearer and more realistic samples, it is not suitable for processing discrete text data. Moreover, it also suffers from training instability, gradient disappearance, and mode collapse. In short, the above-imbalanced treatment methods either have no obvious data enhancement, or the processing process is complex and unstable.

In this work, we propose a novel oversampling algorithm named the borderline nearest neighbor synthetic minority oversampling technique (BNNSMOTE) in response to the previous issues. Our study adopts the fusion algorithm of BNNSMOTE and 1D-MobileNet to handle the data imbalance problem, resulting in higher accuracy, fewer parameters, and lower computing complexity. The specific contributions of this paper can be summarized as follows:

- We use channel screening to improve the operation efficiency and perform data segmentation based on sliding windows to obtain enough samples.
- We introduce data augmentation algorithm BNNSMOTE, for getting more balanced EEG data of epilepsy. Using the idea of the nearest neighbor, the method constructs difficult-to-learn boundary seizure samples after filtering out noise samples and then selects seizure samples at random to be used in the synthesis of new samples. Moreover, we also compared the existing ROS, SMOTE, BLSMOTE, and SVM SMOTE algorithms in detail to reflect the superiority of this algorithm.
- We train a dichotomous 1D-MobileNet model based on seizure detection and compared the parameters and computational load with the traditional network model, which highlights the lightweight characteristics of the model.
- In order to prove the universality of our proposed algorithm, we also use other data sets for verification. We can still get good results on the Bonn dataset, which also proves the generalization ability of our proposed algorithm and model.

Experimental results suggest that our algorithm can significantly improve the binary classification results of epilepsy seizure and nonseizure when compared to conventional imbalanced EEG data processing (IEDP) algorithms, which dramatically enhance the performance of epilepsy detection.

## 3. Proposed Methods

This paper extracts the synchronization features of multichannel epilepsy EEG signals based on EEG signal characteristics and makes various patients train and test separately. In addition, due to the differences between the data of each channel, the signal characteristics contained in them may be complementary, so they should be trained individually while undertaking epilepsy detection tasks. The workflow of the proposed seizure detection system is shown in Figure 1. Raw EEG signals are preprocessed and channel selected before imbalance processing. Next, the processing data are used as 1D-MobileNet input data, which is then trained and tested to identify epilepsy automatically.

### 3.1. BNNSMOTE

In the process of synthesizing new samples, not all seizure samples are important, as some of them may be easily learned and provide little information for the synthesis of new samples. Therefore, it is necessary to identify a sample set of seizures that are difficult to learn and synthesize new samples from them. These samples are usually located near the decision boundary. Although the BLSMOTE algorithm tries to find a set of hard-to-learn samples, it cannot correctly identify all of them. Besides, the BLSMOTE algorithm cannot effectively distinguish noise samples, it will also make the model overlearn boundary data features while weakening other data features. Moreover, in some cases, it does not find seizure samples at borderline locations. To overcome the challenges mentioned previously, we propose a BNNSMOTE algorithm for constructing boundary samples based on the nearest neighbor. This algorithm uses the nearest neighbor notion to generate nonseizure samples near the boundary after filtering out noise samples. Moreover, it identifies the difficult-to-learn seizure samples at the border and lastly selects seizure samples at random to be used in the synthesis of new samples. The basic ideas are as follows:

- We filter the original seizure samples to remove noise
- We construct the hard-to-learn boundary seizure sample set
- We synthesize new seizure samples

Figure 2 shows a schematic diagram of its new sample synthesis.  Algorithm 1 depicts the whole algorithm for augmenting data with BNNSMOTE.

### 3.2. 1D-MobileNet

The existing neural network structure has a big memory need and a huge number of parameter calculation, making it difficult to use on mobile terminals and embedded devices. Based on this, in view of the characteristic that EEG signals are one-dimensional signals, we design a lightweight 1D-MobileNet model. As shown in Figure 3, it includes a one-dimensional convolutional layer (Conv1d), a bottleneck block, an average pooling layer (Average Pooling), a fully-connected layer (FC Layer), and a linear classifier (Linear).  Table 1 shows the model's detailed network parameters, where *t* is the expansion factor, *c* is the channel of the output matrix, *n* is the number of module repetitions, and *s* is the step size.

The core part of the model is the bottleneck block, which includes a depthwise separable convolution and an inverted residual module. Unlike ResNet, the inverted residual always extracts features using depthwise convolution. The difference between it and standard convolution is that the parameters and amount of calculation are substantially reduced when the accuracy is practically unchanged.

## 4. Experiments and Discussion

### 4.1. Dataset

The CHB-MIT EEG dataset, which includes scalp EEG (sEEG) recordings of 23 patients with medically intractable focal epilepsy obtained from 22 subjects, was used in this study [32]. The case “chb24” was added later, and each EEG recording contained 23 commonly used channels [33]. Because the acquisition time of case “chb04” is too long, the duration of case “chb06” and case “chb16” episodes is too short, and case “chb12” comprises alterations in electrode montage. The previous 4 cases will be eliminated in the follow-up study.

### 4.2. Data Processing

It is required to denoise the original signal for the sake of extracting EEG signal features more effectively. This paper filters with a 0.5–50 Hz Butterworth bandpass filter before performing sliding segmentation. In order to increase the amount of samples, we adopt the sliding window of 4 s and the step size of 2 s to select the EEG signal of patients for analysis, with each segment corresponding to 1024 sampled data. The EEG signal of patients is classified into two categories in this paper: ictal and nonictal.

In order to optimize the channel selection, for the 23 commonly used channels, a one-way analysis of variance (ANOVA) was utilized to judge if there is a significant difference between the ictal and nonictal states of the channel. After the previous screening and according to the common channels among different patients, 10 channels were finally determined, as shown in Table 2.

### 4.3. Evaluation Metrics

The detection of seizures is classified as a binary classification problem. In this paper, positive samples represent epileptic seizures, and negative samples represent nonseizures.  Table 3 shows the confusion matrix, which lists the four possible detection results: true positive (TP), false positive (FP), true negative (TN), and false negative (FN) [14]. Equation (1) has a formula for accuracy, equation (2) shows for recall, and equation (3) represents precision.

The F1-score formula as shown in equation (4) is the harmonic mean of precision and recall as follows:

(1) $$\begin{array}{c} Accuracy=\frac{TP+TN}{TP+FP+FN+TN}\text{,} \end{array}$$

(2) $$\begin{array}{c} Recall=\frac{TP}{TP+FN}\text{,} \end{array}$$

(3) $$\begin{array}{c} Precision=\frac{TP}{TP+FP}\text{,} \end{array}$$

(4) $$\begin{array}{c} F1=\frac{2\times precision\times recall}{precision+recall}\text{,} \end{array}$$

A 5-fold cross-validation method was utilized for each situation to evaluate the robustness of the proposed algorithm, which greatly improves its generalization ability. The EEG dataset for each case was separated into two pieces at random in an 8 : 2 ratio. The IEDP technique processes just 80% of the fragments, with the remaining 20% acting as the test set.

### 4.4. Result Analysis

The data set is processed by ROS, SMOTE, BLSMOTE, SVM SMOTE, and BNNSMOTE algorithms, respectively, and the processed data are input into the 1D-MobileNet model for classification and testing. The following is a brief description of several IEDP technologies.

#### 4.4.1. ROS

ROS is the simplest oversampling technique to balance the imbalance of data sets. It balances the data by copying a few class examples without any loss of information. However, if noisy samples are selected for replication, the interference of noise signals will be increased. In addition, too many repeated samples will reduce the decision-making area of the model and cause overfitting.

#### 4.4.2. SMOTE

SMOTE works by using the k-nearest neighbor algorithm to create synthetic data. It can get the new sample data after some operation between the selected two samples and add the new data to the sample data set, which solves the problem of learning repeated feature information from a large number of the same data caused by ROS. However, the SMOTE algorithm cannot effectively solve the effect of noise data on classification. On the contrary, if there are too many noisy data in the data set, the SMOTE algorithm will also synthesize new sample data according to the algorithm principle and add it to the data set. This will aggravate the adverse effect of noisy data on the classifier, thus affecting the overall classification performance.

#### 4.4.3. BLSMOTE

In the BLSMOTE technique, only seizure samples near the boundary were oversampled. It avoids the bad effect of expanding noisy data on the classifier. At the same time, the boundary feature information between the two types of data is strengthened, which makes it easier for the classifier to learn more distinct features from the boundary of the two types of data. However, it cannot effectively distinguish the noise samples and will cause the model to overlearn the boundary data features so as to weaken the influence of other data on the model. Furthermore, in some cases, this method cannot accurately find the seizure samples at the boundary locations.

#### 4.4.4. SVM SMOTE

Another variant of BLSMOTE is SVM SMOTE. This technique combines a support vector machine (SVM) algorithm to identify misclassified points. After training the SVM classifier on the original training set, the boundary region is approximated by the support vector. Synthetic data are then randomly created along a line connecting each seizure sample support vector to its multiple nearest neighbors. However, it has similar pitfalls as BLSMOTE and is difficult to implement for large training samples.

Figure 4 shows the performance effect of different IEDP algorithms in each channel using the channel of case “chb01” as an example. Because each channel carries a varied quantity of information, each channel's accuracy varies, with channel “ch22” having the best effect and the most obvious features. Except for the higher recall rate after SMOTE processing, almost all other indicators have the best effect of BNNSMOTE. Generally speaking, the precision and the recall have an inverse relationship: the greater the precision, the lower the recall; the lower the precision, the higher the recall. Different detection tasks have different requirements for the two. The comprehensive F1-score is commonly used to measure both when there are high criteria for both. Moreover, the higher the F1-score, the more robust the model is. In our paper, in addition to detecting the generally used accuracy, the comprehensive F1-score can better reflect the performance of the algorithm.  Table 4 shows the accuracy and F1-score of the 1D-MobileNet model in each patient. The average accuracy and F1-score of our proposed algorithm achieve the best values of 99.40% and 91.90%, respectively.

Figure 5 shows the detection performance of different IEDP algorithms in every patient. Similar to Figure 4, for almost every case, the proposed algorithm performs best overall in seizure detection. Especially in case “chb09,” her performance metrics have reached the best, with a recall rate of 94.71%, a precision of 100%, an F1-score of 97.62%, and an accuracy of 99.93%. However, there are also some cases with low detection results. For example, the F1-score of case “chb15” after employing numerous IEDP algorithms are 73.4%, 75.86%, 69.31%, 73.66%, and 82.0%, respectively. It is possible that too much noise interfered with the data during collecting, blurring the lines between different sorts of samples. These situations will be improved in future studies to better identify the boundaries between different sorts of samples.

To verify the superiority of our algorithm, we compare the traditional ROS, SMOTE, BLSMOTE, and SVM SMOTE algorithms, as shown in Table 5. The results reveal that after balancing treatment, the detection effect is greatly improved. The SMOTE algorithm has the best recall value but the lowest precision value when compared to unprocessed data. Yet the BNNSMOTE algorithm proposed in this research has the best effect in terms of precision, F1-score, and accuracy. Because the algorithm can not only effectively identify and remove noise samples but also selectively learn seizure samples, identify difficult-to-learn seizure samples, and synthesise new samples to enhance the difference between different samples. The proposed algorithm corrects the flaws in the BLSMOTE algorithm, increasing precision and F1-score by 12% and 6%, respectively. As a result, the overall effect of our proposed BNNSMOTE algorithm is the best, and it outperforms the existing IEDP technique.

Table 6 compares the parameters and computation quantity of several network models. The parameters and calculation amount of the 1D-MobileNet model proposed in this work are only 2.2 M and 94 M. Compared with the traditional network, our network considerably reduces the parameters and calculation amount when the accuracy is improved. Furthermore, the parameters of our model are just half of those in the standard MobileNet model, which is better suited to mobile terminals and embedded devices.

In order to verify the universality of the proposed algorithm, Table 7 shows the comparison of the results of the Bonn dataset after IEDP. No matter what the imbalance ratio between the seizure sample and the nonseizure sample is, the BNNSMOTE algorithm can achieve a good effect in accuracy and F1-score, which also proves the generalization ability of the algorithm.

### 4.5. Performance Comparison

Table 8 compares this work to earlier research, all of which were assessed using the CHB-MIT dataset, including methods, the number of patients, and the indicators. The traditional machine learning methods such as linear discriminant analysis (LDA) [34], SVM [21, 35], random forest (RF) [40], and others were used for seizure detection. These approaches yielded accuracy ranging from 89.49% to 96.87%, with the SVM in [35] attaining the highest accuracy of 96.87% but only 72.99% recall. The deep-learning approaches, including long-short term memory (LSTM) [36, 42], CNN [37, 41], recurrent neural network (RNN) [38], as well as autoencoders [39], achieved the accuracy ranging from 84.00% to 99.83%. Among them, [41] introduced a new model, ScoreNet, which was combined with CNN to obtain the maximum accuracy of 99.83% but only 76.54% recall. In addition, DenseNet-LSTM, a new deep-learning hybrid model developed by [42], achieved over 90% of the four basic indicators. However, the network is too complex and the data imbalance is not dealt with in depth. [43] proposed a graph attention network, which fully explored the spatial relationship of different EEG electrodes on the scalp with the self-attention mechanism. The model also adopted focal loss to deal with the data imbalance problem that appeared in seizure detection, and the final results demonstrated the superior performance and stability of the proposed method. However, when they converted EEG signals into two-dimensional graphics, some data features were lost, resulting in incomplete feature information extracted. In this paper, the original one-dimensional EEG signal is directly input, and all the features are preserved. Different from previous methods, [44] first mixed unsupervised learning (UL) and supervised learning (SL) methods in the field of seizure detection. The hybrid method used a small amount of labeled data to train the model while achieving satisfactory seizure detection performance. Nevertheless, the use of the EasyEnsemble algorithm in undersampling will lead to the loss of sample information during a seizure, ignoring many pieces of potentially useful seizure sample information.

In comparison to the approaches described previously, our algorithm has a 99.40% average accuracy after 5-fold cross-validation, and the recall, precision, and F1-score reach 87.46%, 97.17%, and 91.90%, respectively. Therefore, in terms of accuracy, the performance of our method surpasses most of the previous research in Table 8, demonstrating that the proposed BNNSMOTE and 1D-MobileNet combination was effective. We also had considerable success when we used the Bonn dataset for verification. In fact, the data processing portion of the experiment will take a long time, and a large number of experiments will be required to discover the best outcome. In this work, we used a sliding window of 4 s and a step size of 2 s to expand the data and enhance the diversity of samples and used the 5-fold cross-validation approach to get good results finally. Furthermore, as shown in Table 6, the parameters and calculation amount of the model introduced in this study were greatly decreased compared with other models, saving the system memory. This is not observed in other algorithm models, which is also a major feature of this paper, and it will substantially facilitate the future use of mobile terminals and the realization of embedded AI.

## 5. Conclusions

In this work, we have proposed a novel oversampling method named the BNNSMOTE algorithm for data augmentation to address the imbalance problem in seizure detection. Then, the 1D-MobileNet model was utilized to verify the performance of the proposed algorithm, and the parameters and calculation of the model are greatly reduced. Experimental results demonstrated that this method has a better effect on the CHB-MIT dataset than the existing seizure detection algorithms, which also provides a very effective method for other fields. Such a lightweight network structure also provides a theoretical basis for the development of smart medical care. In the future, on the one hand, it is necessary to improve the effect of data processing, continue to optimize the model algorithm, and enhance the detection performance. On the other hand, it will be combined with embedded hardware to realize embedded AI and truly achieve the purpose of real-time monitoring and real-time alarm.

## Figures and Tables

**Figure 1:** The workflow of the proposed seizure detection system.

**Figure 2:** BNNSMOTE algorithm schematic diagram.

**Figure 3:** 1D-MobileNet model.

**Figure 4:** Performance of using different IEDP algorithms in each channel.

**Figure 5:** Performance of seizure detection using different IEDP algorithms.

**Algorithm 1:** BNNSMOTE algorithm.

**Table 1:** Detailed network parameters of the model.

Input	Operator	*t*	*c*	*n*	*s*
1024 × 1	Conv1d	—	32	1	1
512 × 32	Bottleneck	1	16	1	1
512 × 16	Bottleneck	6	24	2	2
256 × 24	Bottleneck	6	32	3	2
128 × 32	Bottleneck	6	64	4	2
64 × 64	Bottleneck	6	96	3	1
64 × 96	Bottleneck	6	160	3	2
32 × 160	Bottleneck	6	320	1	1
32 × 320	Conv1d 1 × 1	—	1280	1	1
32 × 1280	Avg pool 1d	—	—	1	—
1 × 1280	Linear	—	2	—	—

**Table 2:** Channels retained after channel selection.

Number	Channel
Ch03	T7-P7
Ch04	P7-O1
Ch07	C3-P3
Ch08	P3-O1
Ch13	FP2-F8
Ch14	F8-T8
Ch15	T8-P8
Ch16	P8-O2
Ch20	T7-FT9
Ch22	FT10-T8

**Table 3:** Confusion matrix.

		True condition	
		Seizure	Nonseizure
Predicted condition	Seizure	TP	FP
	Nonseizure	FN	TN

**Table 4:** Results of the 1D-MobileNet model in each patient, on accuracy, and on F1-score.

Patient	Accuracy (%)						F1-score (%)					
	Before	ROS	SMOTE	BLSMOTE	SVMSMOTE	BNNSMOTE	Before	ROS	SMOTE	BLSMOTE	SVMSMOTE	BNNSMOTE
chb01	99.70	99.73	99.12	99.70	99.41	99.81	94.45	95.44	85.08	95.18	90.63	96.22
chb02	99.39	99.36	99.56	99.68	99.45	99.81	89.10	88.44	93.19	94.71	90.46	95.08
chb03	99.53	99.60	98.76	99.52	99.49	99.77	89.96	92.28	82.14	92.24	90.74	94.14
chb05	98.28	99.23	98.43	98.93	99.07	99.51	92.04	92.56	83.77	90.69	91.18	94.33
chb07	99.55	99.59	98.67	99.39	99.21	99.75	90.75	93.64	82.78	91.32	88.56	95.00
chb08	98.72	98.58	96.61	98.70	97.64	99.03	90.24	90.75	71.82	88.27	85.97	94.01
chb09	99.36	99.68	99.91	99.89	99.69	99.93	96.30	94.75	97.28	96.92	95.08	97.62
chb10	99.49	99.52	98.67	99.53	99.39	99.62	89.12	89.79	78.05	90.16	87.59	93.43
chb11	98.64	97.21	96.85	98.08	96.19	98.67	87.02	88.87	85.05	89.32	85.29	93.10
chb13	98.73	98.69	95.48	97.56	95.86	99.00	75.81	79.23	79.29	80.29	75.24	86.04
chb14	98.35	99.28	98.78	98.56	98.38	99.54	80.24	78.22	82.41	83.33	85.00	90.41
chb15	96.98	97.48	93.41	95.53	93.66	97.56	73.41	75.86	69.31	68.43	73.66	82.00
chb17	98.22	98.53	94.48	98.64	98.53	99.23	72.06	83.65	64.03	81.48	78.75	89.42
chb18	99.67	99.67	98.89	99.58	99.25	99.73	89.88	91.93	75.51	85.96	83.25	91.93
chb19	99.70	99.58	99.47	99.77	99.41	99.84	89.42	92.51	91.75	94.36	90.07	94.76
chb20	98.11	99.43	99.24	99.33	99.24	99.56	88.25	90.91	88.10	91.59	88.75	94.62
chb21	98.98	99.25	96.41	98.80	98.77	99.24	78.04	80.28	62.79	64.52	72.04	85.07
chb22	99.44	99.46	99.17	99.51	99.38	99.77	88.34	88.81	82.92	87.52	86.99	94.68
chb23	99.20	99.29	98.05	98.76	98.71	99.29	78.78	85.06	73.11	78.04	76.17	89.06
chb24	98.99	99.05	97.21	98.74	98.83	99.25	80.86	82.43	71.31	75.31	70.32	87.00
Average	98.95	99.11	97.86	98.91	98.48	99.40	85.70	87.77	79.98	85.98	84.29	91.90

**Table 5:** Detection results of different IEDP algorithms.

Method	Rec (%)	Pre (%)	F1 (%)	Acc (%)
Before	78.59	94.55	85.70	98.95
ROS	82.21	94.75	87.77	99.11
SMOTE	90.53	72.15	79.98	98.36
BLSMOTE	87.94	85.04	85.98	98.91
SVMSMOTE	82.18	87.09	84.29	98.48
BNNSMOTE	87.46	97.17	91.90	99.40

**Table 6:** Comparison between different models.

Model	Parameters (M)	Mult-adds (M)
AlexNet	60	720
VGG 16	138	15300
GoogleNet	6.8	1550
ResNet	25.6	3530
Inception V3	23.2	5000
MobileNet	4.2	569
1D-MobileNet	2.2	94

**Table 7:** Performance of different data sets with different IEDP algorithms.

Dataset	Imbalance ratio	Accuracy (%)						F1-score (%)					
		Before	ROS	SMOTE	BLSMOTE	SVMSMOTE	BNNSMOTE	Before	ROS	SMOTE	BLSMOTE	SVMSMOTE	BNNSMOTE
CHB-MIT	1 : 30	98.95	99.11	97.86	98.91	98.48	99.40	85.70	87.77	79.98	85.98	84.29	91.90
Bonn	1 : 4	95.86	96.15	95.60	96.77	96.36	98.30	88.75	89.74	89.01	91.77	90.48	92.11

**Table 8:** Comparison of multiple approaches' experimental results on the CHB-MIT dataset.

Authors	Year	Methods	Patients	Rec (%)	Pre (%)	F1 (%)	Acc (%)
Khan et al. [34]	2012	Multiple wavelet scales, LDA	5	83.6	86.7	85.1	91.8
Janjarasjitt [35]	2017	Wavelet based features, SVM	24	72.99	—	—	96.87
Yao et al. [36]	2018	Attention, BiLSTM	23	87.30	88.29	87.74	87.80
Wei et al. [37]	2019	MIDS, WGANs, 1D-CNN	24	72.11	—	—	84.00
Yao et al. [38]	2019	Windowing, IndRNN	24	88.80	88.69	88.71	88.70
Yuan et al. [39]	2019	STFT-mConvA	23	85.00	85.68	85.34	94.34
Hu et al. [40]	2020	K-means SMOTE, RFS + extra-trees + GBDTs	22	—	—	85.81	89.49
Jiang and Zhao [21]	2021	SMOTE + TomekLink, CSL + SVM	22	86.34	—	—	94.00
Boonyakitanont et al. [41]	2021	CNN, ScoreNet	24	76.54	64.74	70.15	99.83
Ryu and Joe [42]	2021	DWT, DenseNet-LSTM	24	92.92	91.71	92.30	93.28
Zhao et al. [43]	2021	GAT, focal loss	23	97.10	99.59	98.33	98.89
Guo et al. [44]	2022	Isolation forest, time-frequency feature, and easyensemble	24	95.55	—	—	92.62
This work	2022	BNNSMOTE, 1D-MobileNet	20	87.46	97.17	91.90	99.40

LDA: linear discriminant analysis, MIDS: merger of the increasing and decreasing sequences, WGANs: Wasserstein generative adversarial nets, IndRNN: independently RNN, mConvA: multiconvolutional autoencoder, GBDTs: gradient boosting decision trees, CSL: cost-sensitive learning, DWT: discrete wavelet transform, and GA T: graph attention network.

## Data Availability

The CHB-MIT Scalp EEG database is available at https://physionet.org/content/chbmit/1.0.0/(published on 9 June 2010).
